# Process Optimization for Development of Guar Gum-Based Biodegradable Hydrogel Film Using Response Surface Methodology

This article has been retracted.

**DOI:** 10.1155/2022/9180000

**Published:** 2022-08-16

**Authors:** Junaid Aman, Navin Chandra Shahi, Umesh Chandra Lohani, Divya Balodhi, Rajat Singh, Naveen Kumar, Mohd Ishfaq Bhat, Avvaru Praveen Kumar

**Affiliations:** ^1^School of Applied and Life Sciences, Uttaranchal University, Dehradun 248007, India; ^2^G.B. Pant University of Agriculture and Technology, Pant Nagar (US-Nagar) 263145, Uttarakhand, India; ^3^Delhi Technological University, Shahbad Daulatpur, Rohini, Delhi 110042, India; ^4^Department of Food Technology, Khem Singh Gill Akal College of Agriculture, Eternal University, Baru Sahib 173101, HP, India; ^5^Amity Institute of Biotechnology, Amity University, Rajasthan, Jaipur 303002, India; ^6^Department of Applied Chemistry, School of Applied Natural Science, Adama Science and Technology University, P O Box 1888, Adama, Ethiopia

## Abstract

In the current study, a guar-gum-based biodegradable hydrogel film was prepared using an initiator (potassium persulfate), crosslinker (N-N methyl bis acrylamide), and plasticizer (glycerol) for packaging of fruits and vegetables. The effect of independent variables (initiator, crosslinker, and plasticizer) on the biodegradation (% wt. loss), color difference (ΔE), hardness (N), swelling index (%), and transparency (%) of the film was studied using Box–Behnken design, random surface methodology (RSM). The results showed significant effects on all the abovementioned parameters, and it was observed that the developed model was accurate, with a prediction error of only −3.19 to 2.99%. The optimized formulation for the preparation of hydrogel film was 0.15% initiator, 0.02% crosslinker, and 2.88% plasticizer exhibiting satisfactory biodegradability, color difference, hardness, swelling index, and transparency. Results showed that a guar-gum-based biodegradable hydrogel film has adequate physical, optical, and biodegradable properties and can be successfully utilized in the food packaging industry.

## 1. Introduction

In today's world, the industrial symbiosis within the synthetic plastic supply chain results in an increasing volume of nonbiodegradable trash, such as packaging bags, plastic bags, and synthetic polythene, which are hazardous, and cannot be recycled or reused [1–4]. Due to high transparency, softness, low cost, and good barrier properties, plastics were recommended as the most important packaging material. Indeed, excessive use of plastic in food has raised serious environmental and food safety issues [5, 6]. The recycling and incineration of plastic products possess technical and logistic problems [7].

Biodegradable/bioplastic has similar qualities to regular plastic, and it serves a variety of vital functions, such as containment, protection, and quality control [8]. Biodegradable plastics are easily decomposed by the action of microorganisms into the water, carbon dioxide, and biomass. Biodegradable plastics are commonly produced with help of renewable materials, microorganisms, and petrochemicals. The poly-hydroxyalkonates, starch, cellulose, proteins, and polylactic acid are some common examples of biodegradable plastic [9]. These plastics aid in carbon emission reduction, resulting in a significant reduction in the greenhouse effect. It gives an environmentally acceptable answer as well as a long-term future for our planet [10]. However, when biodegradable polymers were explored for use, they revealed several performance and processing issues, including brittleness and temperature of heat distortion, respectively [11]. Extensive research is ongoing in the development of biodegradable packaging films containing various bioactive agents that can enhance the nutritional and sensory properties of fresh food commodities. However, the preparation of biodegradable hydrogels is trending and has gained much attention for the preparation of bio-plastics due to their important polymerization properties [2, 12]. Hydrogel films are superabsorbent by nature, and their manufacturing costs are far lower than synthetic polymers [13]. Hydrogels have a variety of applications including agriculture [14, 15] chemical and biosensors [16], water purification, removal of oil and metal ions [17–19], and medical as well as in food packaging [20]. The creation of poly-ion complex hydrogels is a new way of generating bio-based polymers for food packaging. The production of hydrogels, particularly from natural gums, is attracting attention because it is widely assumed that crude materials will only be available in the near future. The potential uses of natural gum polysaccharides in numerous aspects of food, environment, and medicine industries [21–23]. Guar gums are well-known for their availability, distinctive rheological qualities, and structural variety, in addition to their widespread use in cuisine [10]. Guar gums are a versatile biopolymer produced from plant exudates. Guar gum can absorb a higher amount of water. It should be noted that when compared to gum acacia and other natural gums like xanthan gum and CMCC, guar gum has increased swelling strength [24]. Natural gum-based hydrogels are easy to modify chemically and have several advantages, including the ability to combine with various ceramics and synthetic polymers. Low starch efficiency in terms of water sensitivity, limited mechanical characteristics with high fragility, chemical changes, and even reactions in the active packing of food components are all factors to consider, hydrogel polymerization could not be successfully envisioned.

Hence, considering the abovementioned advantages the present study was carried out to develop a guar-gum-based biodegradable hydrogel film for the packaging of food and other products. The films were prepared using an initiator (potassium persulfate), crosslinker (N-N methyl bis acrylamide), and plasticizer (glycerol). The concentration of the following ingredients was optimized using the response surface methodology (RSM). It is a useful optimization technique since it aids in the discovery of correlations between many independent and response variables while reducing the number of tests and resource usage. The biodegradation (% wt. loss), color difference (∆E), hardness (N), swelling index, and optical properties (transparency) of the film were studied. The accuracy and reliability of the model were checked for validation of the model. Moreover, the developed film showed good tensile strength and has great potential in the packaging of fruit and vegetables.

## 2. Materials and Methods

### 2.1. Materials

Guar gum, potassium persulfate, N-N methyl bis acrylamide, acrylamide, sodium hydroxide, acrylic acid, and glycerol were procured from the Hi-media Pvt. Ltd. Mumbai, India. The electronic weighing balance (Citizen Scale, CX 220), hot air oven (Veliyath Scientific Industries VS101 A), magnetic stirrer with a hot plate (Citizen Scale, 1500 rpm), spectrophotometer (UV-Vis, double beam, LI-2904, LASANY), Incubator (Orbital shaking incubator, Temp: 5°C–60°C), and digital pH meter (Citizen ID50-01) was used.

### 2.2. Formation of Biodegradable Hydrogel Film

The biodegradable hydrogel film was formed using a casting procedure; the suspension solution was dehydrated in the Petri plate. The solution was prepared by dissolving guar gum (1 g) in 100 mL of distilled water having 0.1 g potassium persulfate. The acrylamide (10 g) solution was added to the abovementioned solution with continuous stirring until the solution reaches gelatinization. After that, 0.08 g of N-N methyl bis acrylamide and 4 mL of glycerol were added. The independent variables such as initiator (0.5–0.15%), crosslinker (0.2–0.08 g/mL), and glycerol (2–6 mL) were selected based on previous research [25] and our preliminary studies (Table 1). The solution was stirred for a further 20 minutes for proper mixing and removal of air bubbles. Film-forming suspension solution (100 g) was cast in the Petri plates (15 cm in diameter) and incubated at 60°C in the oven. The prepared film was allowed to cool and then dried at 30°C for 24–48 h. The dried films were peeled off and used for further analysis.

### 2.3. Characteristics of Guar-Gum-Based Biodegradable Hydrogel Film

#### 2.3.1. Biodegradability of Film

The biodegradability of the film was determined using a plastic container (6 × 6 × 6.5 cm) containing natural organic soil. The prepared hydrogel films were cut down into rectangular pieces (2 × 3 cm) and then dried in a hot air oven at 60°C for reducing the moisture content to zero which will help in finding the percentage of weight loss. After drying, the film was placed on an aluminum mesh and buried in the soil up to 4 cm deep in the abovementioned containers. Then, 20 mL of water was added every day to maintain relative humidity at approximately 40% inside the soil. After 15 days, the film sample was removed from the soil and weighed according to the methodology described [26]. The degree of film degradation was determined after 15 days as the weight loss (WL%) of a buried film using the following equation:

(1) $$\begin{array}{c} \text{Weight Loss}\left(\%\right)=\frac{M_{0}-M_{f}}{M_{0}}\times 100, \end{array}$$

where *M*_0_ = Initial mass of film (*g*) and *M*_*f*_ = Remaining mass of film (*g*) after 15 days.

#### 2.3.2. Color Profile Analysis

The color difference of prepared hydrogel film was determined using a combination of a digital camera, computer and Adobe Photoshop CS 5 software provide a less expensive and easy way to determine the color parameters of food products [27]. The brightness coordinate *L*^*∗*^ was used to assess the whiteness value of a color, which ranges from black at 0 to perfect white at 100. The chromaticity coordinates *a*^*∗*^ determined green when negative and red when positive and the chromaticity coordinate *b*^*∗*^ measured yellow when positive and blue when negative [28]. The ΔE, *a*^*∗*^ and *b*^*∗*^ were used to express color degradation/change value as a single numerical value. The following equations (2)–(4) were used to calculate color indices such as *L*^*∗*^, *a*^*∗*^ , and *b*^*∗*^. The ΔE is defined as the magnitude of total color differences and was calculated using (5). The lightness (*L*), *a,* and *b* values were obtained from the histogram window of Adobe Photoshop CS 5 software.

(2) $$\begin{array}{c} L^{*}=\frac{\text{Lightness}}{255}\times 100, \end{array}$$

(3) $$\begin{array}{c} a^{*}=\frac{240\times a}{255}-120, \end{array}$$

(4) $$\begin{array}{c} b^{*}=\frac{240\times b}{255}-120, \end{array}$$

(5) $$\begin{array}{c} E^{*}=\sqrt{{\left(\Delta L^{*}\right)}^{2}+{\left(\Delta a^{*}\right)}^{2}\;+{\left(\Delta b^{*}\right)}^{2},} \end{array}$$

where *E* = Distance matrix (color difference). *ΔL*^*∗*^ = *L*^*∗*^_standard film_—*L*^*∗*^_sample film_. *Δa*^*∗*^ = *a*^*∗*^_standard film_—*a*^*∗*^_sample film_. *Δb*^*∗*^ = *b*^*∗*^_standard film_—*b*^*∗*^_sample film._

Since *ΔL*^*∗*^, *Δa*^*∗*^, and *Δb*^*∗*^ may be positive or negative while the total color difference is always positive.

#### 2.3.3. Mechanical Properties

The mechanical properties of the film were tested using an Instron Universal Testing Machine (Model MDX, Instron Engineering Corporation, Canton, MA, USA) equipped with a 0.5 kN load cell, according to ASTM method *D* 882–88 as the procedure followed [29]. The puncture test (Rockwell hardness test) uses a 60 kg load on the film and the probe used is a ball indenter having a 1/16-inch steel ball. Each film was chopped into 3 cm × 8 cm rectangular pieces. The machine was set to tensile mode with a 50 mm initial grasp separation and a 50 mm/min crosshead speed. The maximum load (N) was divided by the initial cross-sectional area (m^2^) of the films, and the puncture (TS) was given in MPa. Each sample was tested three times and the average value was used for the determination of the puncture (TS) of the film using the following:

(6) $$\begin{array}{c} T_{S}=\frac{F}{S}. \end{array}$$

In this equation:*T*_*s*_-Tensile strength (MPa). *F*-The maximum tensile force when the sample breaks (N). *S*-Cross-sectional area of the specimen (m^2^).

#### 2.3.4. Swelling Properties

Swelling properties were conducted using a buffer solution of pH 7.4 at room temperature. The dried hydrogels of each gum were weighed and immersed in the solution. Periodically each swollen hydrogel was removed, and excess water was wiped using filter paper and weighed to obtain the relation between swelling ratio and time to determine swelling properties [14]. The swelling ratio was calculated according to the given:

(7) $$\begin{array}{c} S=\frac{W_{1}-W_{s}}{W_{s}}, \end{array}$$

where *S* is the swelling ratio, *W*_1_ (mg) is the weight of swollen gel and *W*_S_ (mg) is the initial weight of the dried hydrogel.

#### 2.3.5. Transparency (Optical Properties)

Transparency of the hydrogels was measured in the visible wavelength range at 550 nm using a UV-visible spectrophotometer [30].

### 2.4. Experimental Design and Optimization

#### 2.4.1. Experimental Design

The surface-response methodology 3 factors 3 levels Box–Behnken experimental design was used to study the effect of the initiator, crosslinker, and glycerol concentration on dependent variables (biodegradation, color difference, hardness, swelling index, and transparency). The levels of the independent variables were defined according to a Box–Behnken design. The 3-level factorial designs proposed by Box–Behnken is formed by combining 2^*k*^ factorial with incomplete block design. Box–Behnken design does not contain any point vertices of the cubic region created by upper and lower limits for each independent variable, which means it reduces the number of required runs. It could be an advantage when the point of corners represents factor-level combinations that are prohibitively expensive and impossible to test because of the physical process constant.

As shown in Table 2, a BBD model had 17 experiments with 5 experimental runs at central locations for three factors with three levels. The analysis of variance was used to determine the lack of fit and the significance of the linear, interaction, and quadratic effects of the independent variables on the dependent variables. For each response, a second-order regression model in (8) was created to represent the relationship between the dependent and independent variables, and the model's goodness of fit was tested.

(8) $$\begin{array}{c} Y=\beta_{o}+\beta_{1}X_{1}+\beta_{2}X_{2}+\beta_{3}X_{3}+\beta_{12}X_{1}X_{2}+\beta_{13}X_{1}X_{3}+\beta_{23}X_{2}X_{3}+\beta X_{2}+\beta_{33}X_{3}{}^{2}, \end{array}$$

where *Y* = response calculated by the model, *X* = independent variables, *β*_o_ = constant, *β*_1_, *β*_2_, and *β*_3_ are linear coefficients, *β*_11_, *β*_22_, and *β*_33_ are square coefficients, *β*_12_, *β*_13_, and *β*_23_ are interaction coefficients.

The experiments were conducted according to the standard run as given in the design generated by Design Expert Software version 11.0.1 to determine the predicted value and study the effect of process variables on the preparation of hydrogel film. The predicted values were obtained by a model fitting technique using the Design Expert Software.

#### 2.4.2. Optimization of the Process

The term optimization has been commonly used in analytical chemistry as a means of discovering conditions at which to apply a procedure that produces the best possible responses [31]. Optimizing refers to improving the performance of a system, a process, or a product to obtain the maximum benefit from it. Among the most relevant multivariate techniques used in analytical optimization is response surface methodology (RSM). The objective is to simultaneously optimize the levels of these variables to attain the best system performance. In the present study, optimization was done to develop guar-gum-based hydrogel film. For this, five responses were taken into consideration, i.e., biodegradation (% wt. loss), color difference (∆E), hardness (N), swelling index, and transparency. After that, the optimized condition was predicted by the model. Actual values needed to be examined after performing the experiments on the optimized conditions. For validation, the accuracy and reliability of the model were checked.

#### 2.4.3. Validation of Regression Models

It is also necessary for RSM that the developed regression models provide an adequate approximation for application in a real system, and there are principally two methods used for the validation, i.e., graphical and numerical methods. Validation was done by calculating the percentage error between the actual data (i.e., experimental data) and the predicted data which was obtained by using Design Expert Software version 11.0.1. By doing this, the accuracy and reliability of the model were analyzed [32]. Percentage error was calculated by the formula shown in

(9) $$\begin{array}{c} \text{Percentage Error}=\frac{\left(\text{Actual value}-\text{Predicated value}\right)}{\text{Actual value}}\times 100. \end{array}$$

### 2.5. Statistical Analysis

The data acquired were subjected to regression analysis to determine a link between independent and dependent variables. A mathematical equation that correlates the response surfaces was used to represent each response. The response was then expressed as a second-order polynomial [33].

(10) $$\begin{array}{c} Y=\beta_{o}+\sum_{i=1}^{n}+\beta_{i}X_{i\;}+\sum_{i=1}^{n}+\beta_{ii}X_{i}^{n}+\overset{n}{\underset{i=1}{\sum }}+\sum_{j=i=1}^{n}+\beta_{ii}X_{i}X_{j}, \end{array}$$

where *β*_*o*_, *β*_*i*_, *β*_*ii*_, *β*_*ii*_  = coefficients. *X*_i_ and *X*_j_ = independent variables (where, *i* = 1, 2, ..., *n* and *j* = 1, 2,…, *n*). *n* = number of independent variables (*n* = 3). *Y* = response

Design-Expert Software version 11.0.1 was used to estimate the ideal conditions of independent variables using 2D contour plots. The validity of the model was assessed using analysis of variance (ANOVA), standard deviation (SD), adequacy of model, test for significance, test for lack of fit, coefficient of determination (*R*^2^), and adjusted coefficient of determination (Adj-R^2^). The mean differences of the samples were compared using a one-way analysis of variance (one-way ANOVA). The comparison of means was deemed statistically significant.

## 3. Results and Discussion

### 3.1. Fitting of the Model

In the present study, experiments were conducted to develop natural gum-based hydrogel film for food packaging. Different independent variables were decided based on preliminary experiments. During the preliminary experiments, it was revealed that the initiator, crosslinker, and glycerol influenced the development of biopolymer-based hydrogel film. Natural gum was used as a basic binding agent or matrix material, potassium persulfate is used as an initiator to start the action of polymerization. Acrylic acid and sodium hydroxide are mixed to be used as a monomer. N-N methyl bis acrylamide is used as a crosslinker to improve the mechanical properties of film and provided good texture to film. Glycerol acts as a plasticizer to promote the flexibility and strength of biopolymer film. Also, curing and drying were done to improve the shelf life of biopolymer-based hydrogel film with constant temperature to make the film free from moisture. Different analysis sources of variation such as lack of fit, *R*^2^, predicted residual sum of square (PRESS) for the models, F ratio, and Prob F were studied to discover the fitting of the RSM mathematical models. The coefficient of determination (*R*^2^) was determined to be between 0.94 and 0.99, which means that at least 94% of predicted values could be matched to actual values. Values of F ratio for parameters (biodegradability, color difference, hardness, swelling index, and film transparency) (1.05, 2.20, 3.58, 5.53, and 5.16) and lack of fit (0.46, 0.23, 0.12, 0.06, and 0.073) showed that the designed model was efficient in predicting the physical properties of the film. Statistics revealed that the mathematical model is a good predictor of biodegradability, color difference, hardness, swelling index, and film transparency for barrier properties of the film, with values of PRESS, F value, and lack of fit indicating that the mathematical model is a good predictor of biodegradability, color difference, hardness, swelling index, and film transparency (Table 3). The projected model of films likewise showed high PRESS values, with coefficients of determination (*R*^2^) ranging from 0.94 to 0.99, showing that the model is also accurate for predicting the properties of the hydrogel film.

The magnitude of the predictor's effect on the response was indicated by the probability of significance of the predictor's coefficient. The nature of the influence is explained by the sign and size of the coefficient. At the linear level, a negative sign suggests a decrease in response as the predictor level rises, whereas a positive sign indicates an increase in response. For a fixed value of the response, a significant negative interaction means that the level of one of the predictors can be increased while the level of the other can be decreased. Positive interaction means that the reaction is lowest at the center point and increases as both variables move away from the center point. A positive coefficient of a quadratic term indicates the minimal reaction at the parameter's center point, and it increases as the parameter level increases or decreases. The greatest response is shown by the negative coefficient of the quadratic term at the center values, and it diminishes as the parameter level increases or lowers. In different parts, the results of the experimental and mathematical analysis of different dependent variables were presented.

### 3.2. Model for Predicting Film Qualities Based on Empirical Data

Fitting the experimental data received by the Box–Behnken design into a second-order polynomial mathematical equation (10) yielded the empirical model, using multiple regression analysis on the experimentally obtained data. The following second-order polynomial equation could be used to fit the model. To explore the link between process variables and response variables using the developed mathematical model equations, 2D contour plots were created between two variables while keeping the other variable constant.

(11) $$\begin{array}{c} \text{Bio degradation}=-28.9230+138.2063X_{1}+459.5156X_{2}+11.79381X_{3}–4175.9166X_{1}X_{2}-34.5237X_{1}X_{3}+27.3450X_{2}X_{3}+37.8800X_{1}{}^{2}–1863.6944X_{2}{}^{2}–1.2335X_{3}{}^{2}, \end{array}$$

(12) $$\begin{array}{c} \text{Colour difference}=93.7735-1094.1224X_{1}–578.7034X_{2}–5.9547X_{3}+3083.0900X_{1}X_{2}-64.8571X_{1}X_{3}+24.0652X_{2}X_{3}+3001.6504X_{1}{}^{2}+98.7496X_{2}{}^{2}–0.2516X_{3}{}^{2}, \end{array}$$

(13) $$\begin{array}{c} \text{Hardness}=107.2843+319.6166X_{1}–447.6388X_{2}+6.6216X_{3}+3741.666X_{1}X_{2}-14.625X_{1}X_{3}+103.5416X_{2}X_{3}+2048.5000X_{1}{}^{2}-5106.9444X_{2}{}^{2}–0.8678X_{3}{}^{2}, \end{array}$$

(14) $$\begin{array}{c} \text{Swelling Index}=203.9579+303.9983X_{1}–4338.1805X_{2}+0.4597X_{3}–1826.6666X_{1}X_{2}-274.0250X_{1}X_{3}+317.3750X_{2}X_{3}+6876.8000X_{1}{}^{2}-27252.2222X_{2}{}^{2}+0.8686X_{3}{}^{2}, \end{array}$$

(15) $$\begin{array}{c} \text{Transparency}=-64.0186+1528.6000X_{1}+714.8611X_{2}+3.1420X_{3}–3050.0000X_{1}X_{2}-30.2500X_{1}X_{3}+10.8333X_{2}X_{3}–4848.0000X_{1}{}^{2}-2827.7777X_{2}{}^{2}+\;0.1512X_{3}{}^{2}. \end{array}$$

### 3.3. Impact of Operating Parameters on the Film's Properties

#### 3.3.1. Biodegradation

At the interactive level, Figure 1 represents the contour plot showing the combined effect of initiator and crosslinker at the optimized point of plasticizer of 2.88 mL/100 mL GS. It indicates that the biodegradation increased by increasing the concentration of the initiator and decreasing the concentration of the crosslinker. This is due to the different number of monomer units bonded together by the action initiator and so less amount of crosslinker is required to link the structure in 3D, which can easily absorb water molecules and then the action of microorganisms gets easier and so the hydrogel can easily get degraded into the soil [34].  Figure 1(b) represents the contour plot between an initiator and the plasticizer concentration at the optimized point of the crosslinker of 0.02 mg/100 mL GS. It indicates that the biodegradation increased by increasing the initiator concentration regardless concentration of plasticizer taken within the range, i.e., by increasing or by decreasing beyond the significant limit the rate of biodegradation decreases. This was due to the different number of monomer units that bonded together by the action initiator and less amount of plasticizer causes the film to brittle structure causes less amount of water molecules to diffuse into the hydrogel film and more amount of plasticizer causes the film to the more elastic and jelly structure that opposes the water interaction and decreases the rate of biodegradability [35].

Also, at the interactive level, Figure 1(c) represents the contour plot between the crosslinker and plasticizer at the optimized point of the initiator of 0.15 mg/100 mL GS. It indicates that the biodegradation increased by decreasing the amount of crosslinker and keeping in range the amount of plasticizer, i.e., by increasing or by decreasing beyond the significant limit the rate of biodegradation decreases. This was due to the different number of polymer units formed after the initiation that bonded together by the action crosslinker and less amount of plasticizer causes the film to brittle structure causes less amount of water molecules to diffuse into the hydrogel film structure and if more amount of plasticizer causes the film to a more elastic and jelly structure which opposes the water interaction and decreases the rate of biodegradability [35].

#### 3.3.2. Color Difference

At the interactive level, Figure 2(a) shows the contour plot between the initiator and crosslinker at the optimum point of plasticizer concentration (2.88 mL/100 mL GS). It is visible from the figure that the minimum value of color was obtained between initiator values 0.12 and 0.16 mg/100 mL GS as the crosslinker was increased. It indicates that the color difference increased by increasing the concentration of the crosslinker and decreasing the concentration of the initiator because the free radicals are present in the film which caused the film to luminous side and increased the color difference [36].  Figure 2(b) shows the contour plot between initiator and plasticizer concentration at the optimum point of the crosslinker (0.02 mg/100 mL GS). This plot shows that the minimum value of color difference was obtained between initiator values 0.12 and 0.16 mg/100 mL GS as the plasticizer was increased. It indicates that the color difference increased with increasing the concentration of plasticizer and decreasing the concentration of initiator reason being the lesser number of free radicals released by the initiator and the film being more transparent due to the high concentration of the plasticizer [37]. Similarly, Figure 2(c) shows the contour plot between crosslinker and plasticizer concentration at the optimum point of the initiator (0.15 mg/100 mL GS). This plot shows the maximum value of color was obtained as the concentration of crosslinker and plasticizer was increased. It was observed as the increased amount of crosslinker uses a greater number of free radicals released by the initiator and proper binding takes place which in turn increased by the action of the plasticizer thus reducing the color difference [38].

#### 3.3.3. Hardness

At the interactive level, a contour plot showing the relationship between initiator and crosslinker on the hardness of developed hydrogel film at an optimum value of plasticizer concentration (2.88 mL) is depicted in Figure 3(a). It indicates that the hardness increases with increasing the concentration of the initiator and decreasing the concentration of the crosslinker. This was due to the different number of monomer units that were bound together by the action initiator and so less amount of crosslinker was required to link the structure in 3D, which can easily absorb water molecules. It displays that while increasing the values of initiator and crosslinker up to a certain limit increased the value of hardness after a particular extent of adding initiator and crosslinker loses the bonding as the matrix material, i.e., the natural gum was fixed so the more initiation and cross-linking takes place and loses the strength and so decreases the hardness of the hydrogel film [39]. Similarly, a contour plot showing the relationship between initiator and plasticizer concentration on the hardness of developed hydrogel film at the optimum value of crosslinker (0.02 mg/100 mL GS) is depicted in Figure 3(b). It displays that the low level of initiator, when plasticizer was introduced in developed hydrogel film was increased, there was the increase in the hardness. But at a high initiator and high level of plasticizer concentration the hardness of the hydrogel film decreased to a particular extent. This indicates that average levels of both parameters were responsible for the maximum hardness of the developed hydrogel film [40]. Also, at the interactive level, a contour plot showing the relationship between plasticizer concentration and crosslinker on the hardness of developed hydrogel film at the optimum value of initiator (0.15 mg/100 mL GS) is depicted in Figure 3(c). It demonstrates that at the low level of crosslinker and plasticizer in the hydrogel film, there was a reduction in the hardness. But increasing the levels of the crosslinker and plasticizer the hardness tends to be increased and the film becomes a little hard. While at the high level of crosslinker and plasticizer hardness gradually increases and made the film brittle [41]. This indicates that range levels of both the parameters were responsible for the best hardness of the hydrogel film for food packaging.

#### 3.3.4. Swelling Index

At the interactive level, contour plot showing the relationship between initiator and plasticizer concentration on the swelling index of developed hydrogel film at the optimum value of crosslinker (0.02  mg/100  mL GS) is depicted in Figure 4(a). It represents that at the low level of plasticizer when the initiator in developed hydrogel film is increased from 0.05 to 0.15  mg/100  mL GS, there was an increase in the swelling index. But at a high-level plasticizer, there was not much increase in the swelling index, as the initiator is increased. Likewise, when the plasticizer was kept at a low level, the swelling index of the developed hydrogel film increased, with an increase in the levels of the initiator. This indicates a low level of plasticizer and high level of initiator were responsible for the maximum swelling index of the developed hydrogel film because of the free radicals produced by the initiator that bind with water molecules and tend the film to swell [42]. Similarly, at the interactive level, a contour plot showing the relationship between plasticizer concentration and crosslinker on the swelling index of developed hydrogel film at an optimum value of initiator (0.15 mg/100  mL GS) is depicted in Figure 4(b). It shows that at the low level of the crosslinker and plasticizer concentration, there was an increase in the swelling index of the developed hydrogel film. But while increasing the levels of the crosslinker and plasticizer concentration the swelling index of the developed hydrogel film decreased due to the high bonding and high plasticizing effect the film was not able to absorb more amounts of water molecules [14]. This indicated that low levels of both the parameters were responsible for the maximum swelling index of the developed hydrogel film.

#### 3.3.5. Film Transparency

At the interactive level, a contour plot showing the relationship between initiator and crosslinker on transparency of developed hydrogel film at the optimum value of plasticizer concentration (2.88 mg/100 mL GS) is depicted in Figure 5(a). It depicts that at the low level of the initiator when the crosslinker in developed hydrogel film is increased; there was a very slow gradual increase in the transparency of the film. But at the high initiator, there was an increase in transparency of the developed hydrogel film, as the crosslinker was increased. Similarly, when the crosslinker was kept at a low level, the transparency of the film increased as the concentration of the initiator increased. Whereas at the high level of the crosslinker, transparency of the hydrogel film was increased, as the level of initiator increased. This indicates that high levels of both parameters were responsible for the maximum transparency of the developed hydrogel film. The results showed that with the increase in initiator and crosslinker contained in the gum solution absorbance of UV light in the hydrogel film increased due to the proper and tight bonding of hydrogel which in turn decreased the transparency of the film [43].  Figure 5(b) depicts a contour plot showing the relationship between initiator and plasticizer concentration on transparency of developed hydrogel film at the optimum value of crosslinker (0.02 mg/100 mL GS). It displays that at the low level of plasticizer when the initiator in developed hydrogel film is increased, there was a slight increase in the transparency of the film. But at the high level of plasticizer, there was a rapid increase in transparency of the film as the initiator level increased. Similarly, when the initiator was kept at a low level, transparency of the developed hydrogel film increased with an increase in plasticizer concentration. Whereas, at the high level of initiator, transparency of the film increases at a very slow rate, with the increase in the level of plasticizer concentration. This indicates that a high level of initiator and in-range level of plasticizer concentration was responsible for the maximum transparency of the developed hydrogel film. An initiator releases free radicals in the film, which blocks the UV light passage, and increased concentration of plasticizer made the film hygroscopic and translucent as glycerol is a thick liquid which in turn reduces the transparency of the film [44].

### 3.4. Optimization and Validation of Hydrogel Film Formulation

The objective of the present study was to optimize the level of independent parameters, i.e., initiator (mg/100 mL GS), crosslinker (mg/100 mL GS), and plasticizer (mL/100 mL GS) for the development of natural gum-based hydrogel film. Numerical optimization of the independent variables was carried out using Design expert 11.0.1 statistical software. All the responses, namely, Biodegradability (%wt. loss), color difference (∆E), hardness (N), swelling index (%), and transparency (%) of developed biopolymer film from natural gum (guar gum) were considered for optimization. The optimization was carried out based on the aforementioned criteria. The most optimal values for the creation of a hydrogel film from natural gum are listed in Table 4.

Regression analysis of actual versus predicted model values was done to validate the accuracy of the model. Actual and predicted model values of responses along with the corresponding percentage error are given in Table 5.

All results for observed values are presented in triplicates.

The low % prediction error of 0.11 to 3.19 indicates the high prognostic ability of RSM and hence, verified the accuracy of the model developed from natural gum-based hydrogel film.

## 4. Conclusion

The optimum formulation of guar-gum-based biodegradable hydrogel film was successfully developed from potassium persulfate (initiator), N-N methyl bis acrylamide (crosslinker), and glycerol (plasticizer) using Box–Behnken design by random surface methodology (RSM). The finding showed that independent variables were found to have a significant influence on all of the response variables, either independently or interactively, based on the response surface plots. The level of guar gum was shown to be the most significant (*p* < 0.05) in the development of the film. The results showed that the optimized formulation for the preparation of hydrogel film was 0.15% initiator, 0.02% crosslinker, and 2.88% plasticizer, respectively. The study revealed that guar-gum-based biodegradable hydrogel film could be used as an alternative to conventional plastic for the packaging of fruits and vegetables.

## Figures and Tables

**Figure 1:** (a) Combined effects of initiator and crosslinker on biodegradation at the optimum value of plasticizer concentration (2.88 mL/100 mL GS). (b) Combined effects of initiator and plasticizer concentration on biodegradation at the optimum value of crosslinker (0.02 mg/100 mL GS). (c) Combined effects of crosslinker and plasticizer concentration on biodegradation at the optimum value of initiator (0.15 mg/100 mL GS).

**Figure 2:** (a) Combined effects of initiator and crosslinker on color difference at the optimum value of plasticizer concentration (2.88  mL/100  mL GS). (b) Combined effects of initiator and plasticizer concentration on color difference at the optimum value of crosslinker (0.02  mg/100  mL GS). (c) Combined effects of crosslinker and plasticizer concentration on color difference at the optimum value of initiator (0.15  mg/100  mL GS).

**Figure 3:** (a) Combined effects of initiator and crosslinker on hardness at the optimum value of plasticizer concentration (2.88 mL/100 mL GS). (b) Combined effects of initiator and plasticizer concentration on hardness at the optimum value of crosslinker (0.02 mg/100 mL GS). (c) Combined effects of crosslinker and plasticizer concentration on hardness at the optimum value of initiator (0.15 mg/100 mL GS).

**Figure 4:** (a) Combined effects of initiator and plasticizer concentration on swelling index at the optimum value of crosslinker (0.02 mg/100 mL GS). (b) Combined effects of crosslinker and plasticizer concentration on swelling index at the optimum value of initiator (0.15 mg/100 mL GS).

**Figure 5:** (a) Combined effects of initiator and crosslinker on transparency at the optimum value of plasticizer concentration (2.88 mL/100 mL GS). (b) Combined effects of initiator and plasticizer concentration on transparency at the optimum value of crosslinker (0.02 mg/100 mL GS).

**Table 1:** Coded and actual values of independent variables.

Independent variables	Notation used	Coded and actual values		
		−1	0	1
Initiator (mg/100 mL GS)	*X*_*1*_	0.05	0.10	0.15
Cross linker (mg/100 mL GS)	*X*_*2*_	0.02	0.05	0.08
Glycerol (mL/100 mL GS)	*X*_*3*_	2	4	6

**Table 2:** Box–Behnken three variables experimental design for development of hydrogel-based packaging film.

Experiment no.	Coded value			Actual value		
	*X*_1_	*X*_2_	*X*_3_	Initiator (mg/100 mL GS)	Cross linker (mg/100 mL GS)	Glycerol (mL/100 mL GS)
1	−1	−1	0	0.05	0.02	4
2	0	0	0	0.1	0.05	4
3	0	−1	1	0.1	0.02	6
4	0	0	0	0.1	0.05	4
5	1	0	1	0.15	0.05	6
6	0	0	0	0.1	0.05	4
7	0	0	0	0.1	0.05	4
8	1	1	0	0.15	0.08	4
9	0	1	1	0.1	0.08	6
10	1	−1	0	0.15	0.02	4
11	0	−1	−1	0.1	0.02	2
12	1	0	−1	0.15	0.05	2
13	−1	1	0	0.05	0.08	4
14	0	0	0	0.1	0.05	4
15	0	1	−1	0.1	0.08	2
16	−1	0	−1	0.05	0.05	2
17	−1	0	1	0.05	0.05	6

**Table 3:** Experimental results of response for the development of hydrogel film.

Expt. no	Independent parameters			Responses				
	Initiator (mg/100 mL GS)	Cross linker (mg/100 mL GS)	Plasticizer (mL/100 mL GS)	Biodegradation (% wt. loss)	Color difference (ΔE)	Hardness (N)	Swelling index (%)	Transparency (per mm thickness) %
1	0.15	0.05	2	14.90	**3.97** ^*∗*^	116.8	191.46	61.3
2	0.1	0.05	4	13.91	6.99	129.1	125.36	58
3	0.1	0.05	4	12.84	7.54	129.5	110.56	59.4
4	0.1	0.02	6	4.79	6.73	127.25	120.94	56.2
5	0.1	0.02	2	9.84	10.29	126.65	187.23	49.3
6	0.1	0.08	2	**4.32 ** ^*∗*^	5.41	**103.75** ^*∗*^	132.01	56.3
7	0.05	0.05	6	13.44	10.57	128.5	139.71	39.4
8	0.1	0.05	4	11.54	7.45	**130.85** ^*∗∗*^	121.45	59.8
9	0.05	0.02	4	7.79	**25.65** ^*∗∗*^	128	151.08	**19.3** ^*∗*^
10	0.1	0.05	4	12.41	7.32	129.5	110.56	58.4
11	0.05	0.05	2	6.04	25.10	111.45	**89.70** ^*∗*^	26.6
12	0.1	0.08	6	5.83	7.62	129.2	141.89	**65.8** ^*∗∗*^
13	0.1	0.05	4	13.36	6.99	129.95	119.65	58.6
14	0.05	0.08	4	18.34	14.29	106.85	110.56	40.6
15	0.15	0.05	6	8.49	15.39	128	131.86	62
16	0.15	0.08	4	7.63	15.65	123.35	161.91	59.9
17	0.15	0.02	4	**22.13** ^*∗∗*^	8.516	122.05	**213.3** ^*∗∗*^	56.9

^*∗∗*^, ^*∗*^ indicates the maximum and minimum values.

**Table 4:** Optimum values of developed hydrogel film.

Parameters	Optimum values
Initiator (mg/100 mL GS)	0.15
Cross linker (mg/100 mL GS)	0.02
Glycerol concentration (mL/100 mL GS)	2.88
Biodegradation (% wt. loss)	21.49
Color difference (∆E)	5.46
Hardness (N)	122.98
Swelling index (%)	213.44
Film transparency (per mm thickness) %	59.36

^*∗*^GS: Gum solution.

**Table 5:** Validation of developed natural gum-based hydrogel film.

Responses	Predicated values	Actual value	% Error
Biodegradation (% weight loss)	21.4	20.8	2.99
Color difference (∆E^*∗*^)	5.4	5.6	3.19
Hardness (N)	122.9	121.5	1.21
Swelling index (%)	213.4	213.2	0.11
Film transparency (per mm thickness) %	59.3	59.4	0.15

## Data Availability

All the data are included within the article.

## Abbreviations

GS: Gum Solution
CMCC: Crystallography made crystal clear
N-N MBA: N-N methyl bis acrylamide.
